# Functional Characterization of Two Structurally Novel Diacylglycerol Acyltransferase2 Isozymes Responsible for the Enhanced Production of Stearate-Rich Storage Lipid in *Candida tropicalis* SY005

This article has been retracted.

**DOI:** 10.1371/journal.pone.0094472

**Published:** 2014-04-14

**Authors:** Prabuddha Dey, Monami Chakraborty, Maulik R. Kamdar, Mrinal K. Maiti

**Affiliations:** 1 Advanced Laboratory for Plant Genetic Engineering, Advanced Technology Development Centre, Indian Institute of Technology Kharagpur, Kharagpur, India; 2 Department of Biotechnology, Indian Institute of Technology Kharagpur, Kharagpur, India; Woosuk University, Republic of Korea

## Abstract

Diacylglycerol acyltransferase (DGAT) activity is an essential enzymatic step in the formation of neutral lipid i.e., triacylglycerol in all living cells capable of accumulating storage lipid. Previously, we characterized an oleaginous yeast *Candida tropicalis* SY005 that yields storage lipid up to 58% under a specific nitrogen-stress condition, when the DGAT-specific transcript is drastically up-regulated. Here we report the identification, differential expression and function of two *DGAT2* gene homologues- *CtDGAT2a* and *CtDGAT2b* of this *C. tropicalis*. Two protein isoforms are unique with respect to the presence of five additional stretches of amino acids, besides possessing three highly conserved motifs known in other reported DGAT2 enzymes. Moreover, the CtDGAT2a and CtDGAT2b are characteristically different in amino acid sequences and predicted protein structures. The CtDGAT2b isozyme was found to be catalytically 12.5% more efficient than CtDGAT2a for triacylglycerol production in a heterologous yeast system i.e., *Saccharomyces cerevisiae* quadruple mutant strain H1246 that is inherently defective in neutral lipid biosynthesis. The CtDGAT2b activity rescued the growth of transformed *S. cerevisiae* mutant cells, which are usually non-viable in the medium containing free fatty acids by incorporating them into triacylglycerol, and displayed preferential specificity towards saturated acyl species as substrate. Furthermore, we document that the efficiency of triacylglycerol production by CtDGAT2b is differentially affected by deletion, insertion or replacement of amino acids in five regions exclusively present in two CtDGAT2 isozymes. Taken together, our study characterizes two structurally novel DGAT2 isozymes, which are accountable for the enhanced production of storage lipid enriched with saturated fatty acids inherently in *C. tropicalis* SY005 strain as well as in transformed *S. cerevisiae* neutral lipid-deficient mutant cells. These two genes certainly will be useful for further investigation on the novel structure-function relationship of DGAT repertoire, and also in metabolic engineering for the enhanced production of lipid feedstock in other organisms.

## Introduction

Oleaginous microorganisms are capable of producing more than 20% of their dry biomass as storage lipid, which is mostly triacylglycerol [1]. Studies in the past decade have documented that oleaginous microbes are complementary sources (or even superior in few instances) to plant and animals for lipid feedstock required for various applications in food and nonfood industries [2]–[5]. The predominant component of microbial storage lipid is triacylglycerol (TAG), which is a non-polar, water-insoluble ester of glycerol with three fatty acids. TAG molecules are stored in specialized sub-cellular organelles, known as lipid droplets or lipid bodies that are enclosed within monolayer of phospholipids and hydrophobic proteins. Lipid bodies of some oleaginous microbes also contain small proportion of steryl esters. Lipid body structures are also found in plant seeds, and analogous to animal adiposomes. The TAG is a pivotal component in living organisms for lipid homeostasis, which is fundamental to biological membrane systems and signal transduction processes; in addition to its role in storage of energy and carbon required for cellular activities. TAG molecules of lipid bodies may serve to sequester the harmful lipids or unusual free fatty acids that are toxic to the cells. Moreover, the TAG turnover is related to several pathological conditions in animals including human, e.g. obesity, coronary heart disease, hypertriglyceridemia and type-2 diabetes. On the other hand, the TAG metabolism is crucial for plant-pathogen interaction, pollen maturation, seed development and seedling germination in plants; whereas TAG metabolism has important role in starvation, cellular growth and development in microorganisms. Therefore, proper understanding of the TAG metabolism and its role in lipid homeostasis is central to several aspects of basic and applied researches, including healthcare and bioenergy.

The major route to TAG biosynthesis that is conserved in all eukaryotic organisms including yeasts is the acyl-CoA-dependent Kennedy pathway, where the fatty acids are supplied to glycerol molecules as acyl-CoA species. In this pathway, the acyl-CoA:diacylglycerol acyltransferase (DGAT, EC 2.3.1.20) catalyzes the final and committed step to transfer the 3^rd^ fatty acid to the diacylglycerol (DAG) to make TAG. On the contrary, in the acyl-CoA-independent route of TAG formation in mammals, plants and yeasts, the transfer of 3^rd^ fatty acid to DAG occurs from another DAG or phospholipid by separate enzymes. Thus, the DGAT is a key regulatory enzyme associated mainly with the endoplasmic reticulum to pool the carbon and energy flux towards TAG production in eukaryotes. There are at least two known microsomal DGAT family members, DGAT1 (type-1 DGAT) and DGAT2 (type-2 DGAT), which do not share substantial sequence homology, and are proposed to have distinct physiological roles in TAG metabolism in microbes, plants and animals [6]. DGAT1 is a member of the superfamily of membrane-bound O-acyltransferases [7], whereas the DGAT2 belongs to a family that includes acyl-CoA:monoacylglycerol acyltransferase and acyl-CoA:wax alcohol acyltransferase [8]. In contrast to these enzyme families, a soluble form of DGAT has been identified in cotyledons of *Arachis hypogaea* [9] and *Arabidopsis thaliana* [10], and is grouped into the DGAT3 (type-3 DGAT) family. There is another class of DGAT enzymes known as the ‘PDAT family', members of which utilize the acyl group from phosphatidylcholine for the TAG biosynthesis [11], in one of the acyl-CoA-independent routes mentioned earlier. A novel bifunctional DGAT/wax ester synthase (ADP1) from *Acinetobacter calcoaceticus* has been identified, which is responsible for the synthesis of wax esters as the main constituent of storage lipid in addition to a minor amount of TAGs [12].

Orthologues of both DGAT1 and DGAT2 have been found to be widely distributed in plants and animals. Although DGAT2 genes are very common among the fungi and algae, the DGAT1 gene is rare in these microorganisms [6], [13], [14]. Reverse genetic studies in DGAT knock-out mice have demonstrated that the DGAT2 plays a dominant role in TAG biosynthesis in mammals [15]. Expression levels of DGAT2 are also considered to be related to the skin disease psoriasis [16]. Therefore, DGAT2 represents an important therapeutic target for management or treatment of these disorders. In certain plant species, such as castor bean and tung tree (*Vernicia fordii*) DGAT2 plays a role in the selective accumulation of unusual fatty acids into TAG [17], [18]. Overexpression of the *DGAT2* gene in crop plants represents a potential mean of producing novel value-added oils to meet the growing demands from various industries [19]. A number of studies have been carried out to understand the fatty acid biosynthesis and lipid production pathways to alter the quality and quantity of storage lipid in higher plants. Overexpression of key enzymes of the Kennedy pathway (in contrast to the prokaryotic or plastidial pathway responsible for fatty acid biosynthesis) is by far the most successful strategy until now to increase the content of storage lipid in *Brassica napus*, *Arabidopsis thaliana* and *Nicotiana tabacum* [20]–[23].

In recent years, it has been suggested by many researchers that the genetic engineering of key factors of lipid production pathways could be a promising approach to increase the storage lipid content in plant, microalgae and fungi including yeasts for economic production of lipid feedstocks, which may be useful in several applications, such as biodiesel and nutraceuticals. The *DGAT* gene is one such crucial regulatory factor towards TAG accumulation, as explained earlier. Realizing the importance of DGAT enzyme in storage lipid production for various aspects, several scientists all over the world are engaged in biochemistry, molecular biology and biotechnology of this enzyme [6]. Hence, it is indispensable for bioprospecting diverse microorganisms from various ecological niches for DGAT enzymes having novel structure and function, eventually to redesign the TAG biosynthesis pathway in bioreactor for greater yield of lipid feedstock.

There are not many reports on the characterization of the genes encoding for DGAT enzymes in oleaginous yeast species available till date. One DGAT1 from the oleaginous yeast *Yarrowia lipolytica* [24] and a soluble DGAT in another oleaginous yeast *Rhodotorula glutinis* [25] have been studied. To our knowledge, one such published report so far exists on DGAT2 from *Y. lipolytica* [26]. Very recently, we have characterized an oleaginous yeast *Candida tropicalis* isolate SY005 that can produce storage lipid up to 58% under the specific nitrogen-limiting condition (having a C:N ratio of 150∶1), when a drastic (∼22 fold) up-regulation of DGAT-specific transcript was observed unlike the situation for malic enzyme gene [27]. From the transcript profiling data, it was anticipated that different homologues of *DGAT* gene in the *C. tropicalis* might be responsible for the enhanced accumulation of storage lipid during specific nitrogen-stress condition.

Therefore, we aimed to investigate on the molecular nature of the DGAT-specific activity that was responsible for the enhanced production of storage lipid in this particular yeast strain. The present report documents molecular cloning of the two homologues of *DGAT2* gene from *C. tropicalis* SY005 strain followed by bioinformatics analyses and heterologous expression of the cloned genes in neutral lipid-deficient mutant *Saccharomyces cerevisiae* strain H1246. The study reveals that two isozymes - CtDGAT2a and CtDGAT2b, are not only structurally unique among other reported DGAT2s, but characteristically different from each other in predicted protein structures and biochemical functions. The molecular nature of two novel *DGAT2* gene homologues of *C. tropicalis* SY005 strain explains the phenotypic trait for enhanced production of storage lipid enriched with saturated fatty acids in endogenous and heterologous yeast systems.

## Materials and Methods

### Cloning of the CtDGAT2 gene from *C. tropicalis* SY005 isolate

The BLAST analysis was carried out to search for the gene encoding the DGAT-like protein in the *Candida tropicalis* sequences available in NCBI database. Amino acid sequence of the YALI0E32769g protein (a major acyl-CoA dependent DGAT from oleaginous yeast *Yarrowia lipolytica* and an orthologue of *S. cerevisiae* DGAT2 family) was used as the input sequence to find out related protein(s) in *C. tropicalis.* Among the 9 hits obtained through BLAST search within the nonredundant protein database of *Candida* group, the sequence with highest level of amino acid identity with the YALI0E32769g was found to be an uncharacterized hypothetical protein of 569 amino acids [GenBank accession number XP_002546731.1, indicated by black arrow in Figure S1A], belonging to the *C. tropicalis* MYA-3404 strain. This hypothetical protein also contains the domain specific for DGAT, LPLAT and MGAT superfamily protein (Figure S1B).

A set of specific forward and reverse primers (Table S2) was designed on the basis of this hypothetical DGAT2 homologous sequence. A DNA fragment of ∼1.7 kb was amplified by PCR from the genomic DNA of the oleaginous strain *C. tropicalis* SY005 that was available to us. The amplicon was cloned into TA cloning vector (pTZ57R/T) with InsTAclone PCR Cloning Kit (Fermentas, India) using *E. coli* DH10B as the host (Figure S2). The insert DNAs from recombinant plasmids of few randomly selected clones were sequenced.

### Semi-quantitative RT-PCR

Total RNA was extracted from yeast cells grown on four different nitrogen-stress conditions using RNA extraction kit (Qiagen, India) according to the manufacturer's protocol. RNA quantity was determined by O.D. reading at 260/280 nm in a spectrophotometer (Eppendorf Biospectrophotometer), and the quality of RNA was determined by observing the integrity of rRNA bands in 1.2% agarose gel. For RT-PCR analysis, a set of specific primers was designed (Table S2) based upon the nucleotide sequence of the portion flanking the stretch of repeated glutamic acid residues of CtDGAT2 homologues to amplify this particular part of the cDNA, as there is characteristic length-wise difference of six nucleotides between the two homologues. The 1^st^ strand cDNA was synthesized by respective gene-specific reverse primers with the High-Capacity cDNA Reverse Transcription Kits (Applied Biosystems) using 3 µg total RNA as template according to the manufacturer's protocol. Preliminary optimization experiments were carried out to make the RT-PCR semi-quantitative. The exponential phase of PCR was detected between 20 and 28 cycles (data not shown), and subsequently the PCR for 24 cycles were carried out using the 1^st^ strand cDNA prepared from the total RNA extracted at four different nitrogen-stress conditions. The RT-PCR amplicons (80 bp- and 86 bp-specific for *CtDGAT2a* and *CtDGAT2b*, respectively) were subjected to electrophoresis in 12% polyacrylamide gel and visualized under UV trans-illuminator following ethidium bromide staining.

### Bioinformatics analyses

Multiple sequence alignment was conducted using newly isolated two CtDGAT2 proteins along with reported DGAT2 from other organisms by Jellyfish sequence analysis software (http://www.jellyfishsoftware.com/index.htm;jsessionid=12AB643BBE591CBD2D1124E79A274AD4.node2). Hydropathy profiles were analyzed by Kyte-Doolittle method (http://gcat.davidson.edu/DGPB/kd/kyte-doolittle.htm) [28]. Putative functional motifs present in the two isozymes were identified using PROSCAN (http://npsa-pbil.ibcp.fr/cgi-bin/npsa_automat.pl?page=/NPSA/npsa_proscan.html), and transmembrane helices were predicted using TMHMM (http://www.cbs.dtu.dk/services/TMHMM/). The secondary structures of the two CtDGAT2 isozymes were predicted using phyre2 webserver (http://www.sbg.bio.ic.ac.uk/phyre2/html/page.cgi?id=index). Three-dimensional structure of CtDGAT2a and CtDGAT2b were developed using MODELLER 8v2 taking the crystal structure of glyceraldehyde-3-phosphate dehydrogenase from *Methanocaldococcus jannaschii* DSM 2661 (PDB ID: 3RHD) as the template showing sequence identity of >35% with both isozymes revealed by PSI-BLAST [29]. Energy minimization of the resulting model was carried out by Insight II program (version 2000.1, 2000; Accelrys), and the best model was stereo-chemically evaluated by PROCHECK (http://www.ebi.ac.uk/thornton-srv/software/PROCHECK). All the pictorial representations were prepared using PyMol (http://www.pymol.org).

### Preparation of different mutated version of CtDGAT2 gene constructs

Five deletions, 2 replacements and 1 insertional mutation of the *CtDGAT2b* gene were prepared by PCR amplification using specific set of forward and reverse primers (Table S2). The full length *CtDGAT2a* and *CtDGAT2b* genes along with all the mutated versions of the *CtDGAT2b* gene were subcloned individually in the pYES2 plasmid (Invitrogen) for subsequent transformation into the *S. cerevisiae* quadruple mutant (QM) strain (described below). Moreover, the full length *CtDGAT2a* and *CtDGAT2b* genes and few selected mutated versions of *CtDGAT2b* gene were further subcloned separately into pYES2/CT vector (Invitrogen) carrying a C-terminal V5 epitope fused with 6XHis tag to study recombinant protein expression in transformed QM cells of *S. cerevisiae*.

### Strains of *S. cerevisiae* used for transformation

The *S. cerevisiae* BY742 strain was used as the wild-type (WT) yeast. The quadruple mutant (QM) strain H1246 (MATΔ are1-Δ::HIS3, are2-Δ::LEU2, dga1-Δ::KanMX4, lro1-Δ::TRP1 ADE2) of *S. cerevisiae* has knockout mutations for the DGA1, LRO1, ARE1 and ARE2 genes, and thus is defective in TAG and sterol biosynthesis. This QM yeast strain (kindly provided by Dr. S. Stymne, Scandinavian Biotechnology Research, Alnarp, Sweden) was used as the host for heterologous expression of two CtDGAT2 homologous genes and all the mutated versions of CtDGAT2b gene. The QM yeast cells were transformed with either the control (non-recombinant) plasmid or recombinant plasmid carrying the respective gene by the lithium acetate-PEG method using S.C. EasyComp transformation kit (Invitrogen) following the protocol provided in the manual. The transformants were selected on plates lacking uracil and cultivated in yeast nitrogen base (YNB) with 2% (w/v) dextrose. Cells were then harvested, washed with water, and inoculated in induction medium, where dextrose was replaced by 2% (w/v) galactose and 1% (w/v) raffinose to induce the transgene expression.

### Qualitative analysis of lipid

Fluorescence microscopic analyses of the Nile red-stained wild-type (WT) yeast cells and transformed QM cells, harboring either the pYES2 non-recombinant plasmid or recombinant plasmid with the particular gene, were carried out to examine the presence of storage lipid in yeast cells as described previously [30], and the samples were observed under laser-scanning confocal microscope with 488 nm excitation and 585 nm emission filters (Fluo View FV1000 confocal microscope, Olympus). The standard chloroform:methanol extraction procedure was followed for lipid extraction following Bligh and Dyer method [31] with slight modification as described previously [27]. The neutral lipid fractions were resolved by thin layer chromatography (TLC) following the reported method [32] on Silica Gel 60 plates (Merck, Germany) in solvent system of petroleum ether:diethyl ether:glacial acetic acid (70∶30∶1, v/v), and identified by comparing with respective standards.

### Quantitative estimation of total lipid

Both gravimetric measurement [31] and Nile red fluorescence assay [30], [33] were performed to estimate lipid content of wild-type cells, QM cells and QM cells transformed with individual *CtDGAT2* gene construct. Yeast cells were grown on induction medium for 4 days, and biomass was harvested by filtration, and lyophilized to store at −70°C for future use. For gravimetric measurement, lipid was extracted by following Bligh and Dyer method of lipid extraction [31], with slight modification. Briefly, a 50-ml culture sample was centrifuged at 1500 g for 5 min, after which the cells were washed twice with 50 ml of distilled water. Cell pellet was then crushed with liquid nitrogen and the dried biomass was stirred with 20 ml of chloroform:methanol mixture (2∶1) at room temperature for 3 h, followed by centrifugation at 1500 g for 5 min at room temperature to separate the aqueous upper phase and organic lower phase. Next, the lower phase containing lipid molecules was recovered with a Pasteur pipette, and evaporated under reduced pressure for 10 min. The dry lipid samples were weighed.

For Nile red fluorescence assay, yeast cells were grown on induction medium for 4 days. After that, 95 µl cell suspension was taken from each of the culture, and 5 µl Nile red stain was mixed with it, and incubated in dark for 5 minutes. Cell suspension was washed with PBS buffer and the fluorescence intensity was measured before and after addition of Nile red. The first measurement was subtracted from the second measurement, and the results were divided by A_600_ nm with appropriate dilutions. Both types of quantitative estimations were conducted with three individual cultures for each set of experiments and with three replicates.

### *In vivo* fatty acid supplementation assay

The test for cytotoxic effect due to free oleic acid in growth medium was carried out to understand the enzymatic fraction of CtDGAT2b following the method described before [25], with slight modification. Oleic acid was dissolved in ethanol at 0.5 M concentration and later diluted in warm medium with non-ionic surfactant Tween-80 (0.01%, v/v) immediately before yeast inoculation. Wild-type and QM cells were grown on YNB medium with uracil (URA+) and 2% dextrose. On the contrary, the QM strain containing either the non-recombinant pYES2 plasmid or the recombinant plasmid with the CtDGAT2b gene was grown in YNB without uracil (URA-) medium containing 1% raffinose and 2% galactose for the induced expression of the transgene. Different dilutions (10^−1^, 10^−2^, 10^−3^, 10^−4^ and 10^−5^) of yeast cells (with O.D. 1) were plated on oleic acid supplemented media to carry out the experiments.

To determine the fatty acid substrate preference of CtDGAT2b isozyme compared to the endogenous ScDGAT2 of *S. cerevisiae* cells, three different fatty acids like α-linolenic acid (ALA), arachidonic acid (ARA) and erucic acid (EA) were supplemented both in soild and liquid media. Plates of YNB (URA+ or URA-) containing different concentrations of each fatty acid dissolved in ethanol were prepared as described previously [34].

### Preparation of fatty acid methyl esters and determination of fatty acid profiles

Fatty acid methyl ester (FAME) of the neutral lipid fraction of yeast cells grown on different culture conditions was prepared out following the method described earlier [27]. The FAME conversion of each neutral lipid fraction was checked by TLC along with a standard FAME (data not shown). Finally, small volume (3–5 µl) of the prepared FAME sample was analyzed by gas chromatography (PerkinElmer, Clarus 500), fitted with a flame ionization detector and Omegawax-250 capillary column (30 m length, 0.25 mm internal diameter and 0.25 µm film thickness, Sigma). Identification and quantification of individual chromatographic peaks were carried out by means of external standard (Supelco 37-Component FAME Mix, Sigma) and their corresponding calibration curves.

### SDS-PAGE and immunoblotting analysis

Total protein from transformed *S. cerevisiae* cells was isolated using breaking buffer (50 mM sodium phosphate, pH 7.4, 1 mM EDTA, 5% glycerol, 1 mM PMSF) followed by intermittent vortexing with acid-washed glass beads (Sigma-Aldrich, India). For immunoblotting, representative protein samples of equal amount were separated by SDS-PAGE and subsequently electro-transferred onto nitrocellulose membrane. The membrane was then rocked for 2 h at room temperature in blocking solution [PBS buffer supplemented with 0.2% Tween 20 (v/v) and 2% BSA (w/v)]. Chromogenic detection was carried out with Opti-4CN kit (Bio-Rad) after incubating the membrane in appropriately diluted respective primary antibody (1∶4000 for mouse monoclonal anti-His antibody) followed by corresponding secondary antibody (1∶2000 for HRP conjugated anti-mouse, G Bioscience).

## Results and Discussion

In our previous report, while characterizing an oleaginous yeast *C. tropicalis* SY005, differential regulations of two key genes i.e., malic enzyme and DGAT involved in lipid productivity were tested during four different nitrogen-stress conditions [27]. The investigation documented ∼22 fold upregulation of the *DGAT* gene-specific transcript during maximum lipid production stage correlating to a specific nitrogen-stress with the C:N ratio of 150∶1. From the transcript profiling data, it was hypothesized that different homologues of *DGAT* gene in the *C. tropicalis* might be expressed at different stages of its growth or life cycle, and definitely upregulated during specific nitrogen-stress condition for the enhanced accumulation of storage lipid [27].

### Differential expression of two DGAT2 gene homologues under nitrogen-stress condition for enhanced storage lipid production in *Candida tropicalis* SY005 strain

To further understand our previous findings in detail, we cloned and sequenced DGAT-specific gene from this oleaginous yeast. Sequence analysis of the newly cloned insert DNAs revealed the presence of two homologous genes of type-2 DGAT in this strain of *C. tropicalis* (Figure S3), designated as *CtDGAT2a* and *CtDGAT2b* with the GenBank accession numbers KJ437597 and KJ437598, respectively. The *CtDGAT2a* homologue showed 100% nucleotide sequence identity with the reported sequence [XP_002546731.1] of *C. tropicalis* MYA-3404 available in public database, whereas the *CtDGAT2b* is different in 21 nucleotides, resulting in alteration of 9 amino acids (Figure S3). To find out any differential expression of the transcript corresponding to the two CtDGAT2 homologues at four different nitrogen-stress conditions during enhanced storage lipid accumulation, RT-PCR was carried out. Analysis of RT-PCR amplicons showed that the expression of CtDGAT2a homologue was detectable in all four stress conditions, gradually increasing from C:N ratio of 50∶1 to 200∶1 (Figure 1A). On the other hand, the expression of CtDGAT2b isoform was found to be predominant in 150∶1 (C:N) stress condition (Figure 1A), where the lipid accumulation was also observed to be maximum [27]. These results indicated differential expression of two homologues of *CtDGAT2* gene at different nitrogen-stress conditions correlated to the enhanced production of storage lipid in *C. tropicalis* SY005 strain.

**Figure 1:** Identification of two structurally novel CtDGAT2 isozymes in *C. tropicalis* SY005 yeast during storage lipid production. (A) Ethidium bromide-stained 12% polyacrylamide gel of RT-PCR products (80 bp and 86 bp) showing differential expression of two homologous genes, *CtDGAT2a* and *CtDGAT2b* at four different nitrogen-stress conditions i.e., carbon (C):nitrogen (N) 50∶1, 100∶1, 150∶1 and 200∶1. In first two conditions (50∶1 and 100∶1), only the *CtDGAt2a* was found to be expressed, whereas both genes expressed in 150∶1 and 200∶1. Bar diagram represents relative expression of the two CtDGAT2 transcripts, calculated after densitometric scanning of the gel picture. The star indicates undetectable expression of the CtDGAT2b transcript in first two conditions (C:N 50∶1 and 100∶1). (B) Multiple amino acid sequence allignment of both CtDGAT2a and CtDGAT2b isoforms along with other five representatives of DGAT2 reported. Three motifs with remarkable sequence conservation required for DGAT activity found in all DGAT2s are indicated by rectangular box. Two brown colored boxes represent the absence of the critical Cys residue involved in N-ethylmaleimide-mediated enzyme inhibition and the neutral lipid-binding domain FVLF in two CtDGAT2 isoforms with respect to the ScDGAT2. Other colored boxes indicate the presence of five (D1 to D5) unique stretches of amino acids found specifically in two CtDGAT2 isoforms. Five representatives of DGAT2 reported from other organisms are: AtDGAT2, *Arabidopsis thaliana* NP_566952; CeDGAT2, *Caenorhabditis elegans NP_507469.1*; MrDGAT2a, *Mortierella ramanniana AAK84179*; ScDGAT2, *Saccharomyces cerevisiae NP_014888*; VfDGAT2, *Vernonia fordi ABC94474*.

In the past, presence of more than one isoform of DGAT2 has been reported in microalgae *Chlamydomonas reinhardtii*, where five type-2 DGAT homologous genes contribute towards TAG production [13]. Among the plants, although occurrence of *DGAT2* gene has been reported in several species [6], two isoforms of DGAT2 have been documented so far in *Arachis hypogaea* [35]. However, no other reports are available so far except the present study, where more than one homologue of *DGAT2* gene has been characterized in fungus, especially in oleaginous yeast. Although, detail genetics of *C. tropicalis* SY005 strain with respect to the CtDGAT2 gene has not been carried out, it is possible that the *CtDGAT2a* and *CtDGAT2b* homologues could be two alleles of the same gene.

### Two isoforms- CtDGAT2a and CtDGAT2b are unique in primary structure among the reported DGAT2s

To verify *in silico* the DGAT2-specific conserved motifs in the newly cloned isoforms, the amino acid sequences of CtDGAT2a and CtDGAT2b were aligned with homologous sequences of DGAT2 obtained from *Saccharomyces cerevisiae*, *Mortierella ramanniana*, *Arabidopsis thaliana*, *Vernicia fordii*, and *Caenorhabditis elegans* using Jellyfish sequence allignment software. Here five types of different organisms i.e., yeast, mold, model plant, tung tree and nematode were considered as representative organism of species that are evolutionary diverged. Three regions with remarkable sequence conservation are observed amongst all the DGAT2 enzymes (Figure 1B). First, the motif YFP (^129^YFP^131^ in ScDGAT2) is completely conserved (^152^YFP^154^) in the two CtDGAT2 isoforms. Second, the motif HPHG (^193^HPHG^196^ in ScDGAT2) is also conserved (^234^HPHG^237^) in the CtDGAT2a and CtDGAT2b isoforms. The third motif consisting of RXGFX(K/R)XAXXXGXXX(L/V)VPXXXFG(E/Q) spans the longest conserved region in DGAT2-homologous proteins. This motif is found in between the amino acid residues 288 and 311 in ScDGAT2, 394 and 417 in CtDGAT2a, and 396 and 419 in CtDGAT2b. However in ScDGAT2, this motif is in close proximity to Cys^314^ residue, which has been previously demonstrated to be the locus of N-ethylmaleimide-mediated enzyme inhibition. Even though the two CtDGAT2 isoforms are yeast derived, the Cys is replaced by corresponding Val^420^ in CtDGAT2a and Val^422^ in CtDGAT2b, analogous to the situation in DGAT2 of *A. thaliana*. It is noteworthy that a putative neutral lipid-binding domain, FLXLXXXn (where n is a nonpolar amino acid) commonly found in proteins of DGAT2 family including ScDGAT2 (^71^FVLF^74^), is not present in the newly cloned two CtDGAT2 isoforms as well as in *A. thaliana* DGAT2. More interestingly, compared to other reported DGAT2 proteins, there are five unique stretches of amino acids present in CtDGAT2a and CtDGAT2b, designated in this study as D1, D2, D3, D4 and D5 domains (Figure 1B), in addition to the conserved motifs mentioned earlier. A phylogenetic analysis using the amino acid sequences of DGAT2s revealed that the two CtDGAT2 isoforms are intimately related to one another and have close relationship to the DGAT2 proteins from other species of yeasts and fungi, but distantly related to that of other organisms (Figure S4).

Further *in silico* analysis was carried out to investigate the potential structural features of two CtDGAT2 isoforms by comparing the hydropathy profile of DGAT2 proteins from *S. cerevisiae* and *Vernicia fordii*, where topological orientations were experimentally tested [36]. The distributions of sequence motifs in *C. tropicalis*, *S. cereviseae*, and *V. fordii* DGAT2 proteins were analyzed in Kyte-Doolittle hydropathy plots [28]. Although the DGAT2 proteins of three organisms display apparently similar plots, there are characteristic differences (Figure 2). The N-terminal region of each protein contains a hydrophilic stretch followed by a hydrophobic region, except that the hydrophilic tail in VfDGAT2 is significantly shorter. The ScDGAT2 has a continuous sequence of mostly hydrophobic amino acids between 192^nd^ and 250^th^ residues (Figure 2), which contains the conserved motif HPHG (Figure 1B); in contrast, neither of the CtDGAT2 isoform has continuous hydrophobicity in similar region (Figure 2) but HPHG motif is present within both (Figure 1B). Interestingly, both the CtDGAT2 isoforms have other two exclusive hydrophilic regions between residues 250-300 and 350-400 (highlighted by green boxes D3 and D4, respectively in Figure 2), which are not present in DGAT proteins of other two organisms.

**Figure 2:** Comparison of hydropathy profiles of CtDGAT2a and CtDGAT2b with DGAT2s from *S. cerevisiae* and *V. fordii* revealed uniqueness of two CtDGAT2 isozymes. Hydropathy plots were generated by Kyte & Dollite method (28). X-axis and Y-axis indicate number of amino acid residues and hydrophobicity, respectively. Two green outlined boxes (D3 and D4) in CtDGAT2 isoforms indicate the presence of unique hydrophilic stretch of amino acids exclusively present in CtDGAT2.

### CtDGAT2a and CtDGAT2b are characteristically different in amino acid sequences and at the predicted secondary and tertiary protein structure

The derived polypeptide sequences of two newly cloned gene homologues- *CtDGAT2a* and *CtDGAT2b* were analyzed in details using bioinformatics tools to find out any differences between these two at the level of primary, secondary and tertiary protein structure. PROSCAN (http://npsa-pbil.ibcp.fr/cgi-bin/npsa_automat.pl?page=/NPSA/npsa_proscan.html) programme identified five putative functional motifs, and two of these display differences between CtDGAT2a and CtDGAT2b with respect to the position as well as amino acid composition (Table S1).

Analysis of the predicted secondary protein structures using phyre2 program (http://www.sbg.bio.ic.ac.uk/phyre2/html/page.cgi?id=index) revealed the existence of differences between the two isoforms at several positions of α-helices and β-sheets throughout the length of the proteins (Figure 3A). The membrane topology distribution of CtDGAT2a and CtDGAt2b isoforms was evaluated, showing almost the same predicted internal structures. Using TMHMM (TMHMM Server v. 2.0), we identified one potential transmembrane helix at the amino acid position 91–113 (Figure S5), suggesting that these proteins are located in the membrane system. Interestingly, the CtDGAT2b isoform indicates a higher probability of the presence of yet another transmembrane region between the residue numbers of 220–300 compared to CtDGAT2a (Figure S5).

**Figure 3:** Two CtDGAT2 isoforms are different from each other at the level of secondary and tertiary structures. (A) Predicted two-dimensional structure of CtDGAT2a and CtDGAT2b isoforms. Black circles indicate the differences between the two. (B) Three-dimensional structure of two molecular models prepared using MODELLER and validated using PROCHECK. The green model represents the CtDGAT2a, whereas the red model represents the CtDGAT2b. Structural overlapping of the two models created regions A, B, C and D of extra side chain loops, formed by amino acid residues approximately 425–435, 385–430, 450–500 and 365–375, respectively.

Through analysis of the predicted 3-D structures of both CtDGAT2a and CtDGAT2b, four striking differences were clearly visible in the structural overlap of the two models (Figure 3B). Two extra large side chain loops are observed in CtDGAT2a, formed by residues 425–435 and 365–375 as indicated by A and D, respectively. On the contrary, a prominently large side chain loop is formed in CtDGAT2b due to residues 385–430 as indicated by B. Moreover, there is a slight difference between the two isoforms in the orientation of one α-helix that is indicated at the position C, comprising the amino acid residues 450–500 (Figure 3B).

Since two CtDGAT2 isoforms are unique in amino acid sequence compared to the reported DGAT2 proteins, particularly with respect to the five additional domains D1 to D5, we speculated novel biochemical activity of these isoforms in native yeast *C. tropicalis*. Moreover, on the basis of the significant differences in the predicted primary, secondary and tertiary protein structures, we also hypothesized that the two isoforms of CtDGAT2 might have different physiological functions *in vivo*. Hence we constructed two recombinant vectors of pYES2 using *CtDGAT2a* and *CtDGAT2b* genes, and studied the heterologous expression of these two isoforms in neutral lipid-deficient quadruple mutant *S. cerevisiae* H1246 strain to establish their biochemical functions.

### Both the isoforms are functionally active, and the CtDGAT2b isozyme is catalytically more efficient than CtDGAT2a for storage lipid production in heterologous yeast system

Yeast cells usually accumulate TAG and sterol esters during stationary phase of growth in cytosolic lipid bodies [37]. The mutant *S. cerevisiae* H1246 strain, which lacks the genes essential for the formation of TAG (*DGAT* and *PDAT* genes) and sterol esters (*ARE1* and *ARE2* genes), does not form these lipid bodies. Since the activity of at least one of these four genes is sufficient to restore the formation of lipid bodies, we wanted to determine whether lipid bodies could be established in this mutant strain upon expression of the full length CtDGAT2 isoforms.

The transformed *S. cerevisiae* cells harboring the recombinant pYES2 with either *CtDGAT2a* or *CtDGAT2b* gene were induced using galactose, the total protein samples were harvested, and verified through western blotting. Analysis revealed that the two recombinant proteins i.e., the full length CtDGAT2a and CtDGAT2b of predicted molecular mass ∼63kDa gave positive signals on western blot (Figure 4A), confirming the presence of heterologously expressed protein after 6 h of induction. This time period was found to be the optimal incubation time for induction of the recombinant CtDGAT2 proteins in transformed yeast cells.

**Figure 4:** Both CtDGAT2a and CtDGAT2b are functionally active to produce TAG in *S. cerevisiae* QM strain, and the CtDGAT2b is catalytically more active. (A) Western blot showing the recombinant protein of ∼ 63 kDa produced upon galactose induction of yeast QM cells transformed with the full length *CtDGAT2a* or *CtDGAT2b* gene expression cassette prepared in pYES2/CT plasmid. Immunodetection was carried out with mouse anti-His monoclonal antibody. (B) Nile red fluorescence confocal microscopy showing lipid body formation is restored in yeast QM cells upon expression of either CtDGAT2a (QM-CtDGAT2a) or CtDGAT2b (QM-CtDGAT2b). The yeast wild-type BY742 cells were used as positive control (WT), and the QM cells harboring the non-recombinant plasmid was used as negative control (QM-pYES2). (C) Complementation of the TAG-deficient phenotype of the yeast QM strain by expression of either CtDGAT2a or CtDGAT2b. Neutral lipid fractions were separated by TLC, and lipid spots were visualized as described in experimental methods. (D) Bar and line diagrams representing gravimetric measurement and Nile red fluorescence assay of lipid content in QM cells after expression of the full length CtDGAT2a and CtDGAT2b, along with the WT and QM cells transformed with the non-recombinant plasmid as positive and negative controls, respectively. Fluorescence was measured at the stationary phase using 485nm (excitation) and 540nm (emission) before and after the addition of Nile red dye, and expressed in arbitrary unit.

Lipid-specific fluorescent dye Nile red was used to visualize microscopically the presence of lipid bodies in *S. cerevisiae* wild-type (WT), quadruple mutant (QM) cells transformed with the non-recombinant plasmid pYES2 and QM cells expressing either CtDGAT2a or CtDGAT2b. The emission maximum of Nile red conjugated with neutral lipids differs from that of the dye-polar lipid complex. Moreover, the intensity of fluorescence caused by the interaction of the dye with neutral lipid is much higher than that with polar lipid, making Nile red suitable for our purpose of qualitative assessment.

As expected, lipid bodies were detected in the wild-type *S. cerevisiae* cells, but absent from the QM strain harboring only the control plasmid (Figure 4B). However, expression of either CtDGAT2a or CtDGAT2b in QM cells successfully restored the ability to form the neutral lipid bodies (Figure 4B), reflecting the functional activities of both CtDGAT2a and CtDGAT2b enzymes to interact with the *S. cerevisiae* lipid metabolic pathway. Following expression, total lipid extracts from the transformed and non-transformed yeast cells were prepared, and then subjected to thin layer chromatography. Analysis revealed that the TAG could not be detected in QM yeast cells lacking the endogenous DGAT and PDAT activity, whereas the wild-type cells having both the endogenous genes accumulated normal level of TAG as usual (Figure 4C). Upon expression of either CtDGAT2a or CtDGAT2b in QM cells, a prominent spot corresponding to TAG became visible in the total lipid implying a successful restoration of the neutral lipid-deficient phenotype of QM strain by the biochemical activity of either isozyme (Figure 4C). This result indicates that both CtDGAT2a and CtDGAT2b indeed encode an enzymatic activity involved in the biosynthesis of TAG.

To verify which of the isozymes of CtDGAT2 is more efficient i.e., the enzymatic capacity to produce more TAG, we estimated total lipid contents of the transformed yeast cells through Nile red fluorescence spectrometry assay. Lipid-specific Nile red dye moves freely across cellular membrane and thus makes it possible to perform the quantitative neutral lipid assay in living cells, eliminating the need for sample preparation. Moreover, Siloto *et al*. have proved that the DGAT activity can be quantified by Nile red fluorescence spectrometry assay, which is comparable with the standard *in vitro* radioactive assay [34].

Therefore, we also used this simple and reliable fluorescence spectrometry assay after staining with Nile red to quantify the amount of TAG that accumulated in the *S. cerevisiae* wild-type cells, QM cells transformed with the control plasmid pYES2 and QM cells expressing either CtDGAT2a or CtDGAT2b. The fluorescence increase (ΔF) of QM cells expressing each CtDGAT2 isozyme was found to be significantly more than wild-type *S. cerevisiae* cells and extremely high compared to the QM cells harboring the non-recombinant plasmid without the gene of interest (Figure 4D). Estimation showed that the accumulation of TAG is 12.5% more in the QM cells transformed with the *CtDGAT2b* gene compared to that with the *CtDGAT2a* gene. Therefore, the finding elucidated that the isozyme CtDGAT2b is catalytically superior and capable of producing more storage lipid than the CtDGAT2a isozyme.

Previously, the functions of DGAT2 enzymes from three microalgae species, *Ostreococcus tauri*, *Thalassiosira pseudonana* and *Phaeodactylum tricornatum* have been confirmed by restoring the TAG biosynthesis in this neutral lipid-deficient quadruple mutant strain H1246 of *S. cerevisiae* [38], [39], [32]. Among the plants, activities of *Brassica napus* DGAT1 and *Tropaeolum majus* DGAT1 have also been characterized by using the same strain [34], [40].

### The CtDGAT2b is capable of incorporating exogenous fatty acids in TAG, and is having preferential saturated fatty acid specificity in heterologous yeast expression system

The DGAT enzyme can carry out the metabolic channeling of exogenous or unusual fatty acid into TAG, besides incorporating the normal cellular fatty acids into the later. Wild-type *S. cerevisiae* cells grow normally without any growth defect in the presence of unsaturated fatty acids, especially when free oleic acid is in the medium. However, the yeast neutral lipid-deficient QM cells with or without the non-recombinant plasmid exhibit a growth defect in the medium containing free fatty acids. To test whether the CtDGAT2b isozyme is equally efficient in rescuing yeast cells from free fatty acid toxicity, the QM cells transformed with either the non-recombinant or recombinant plasmid carrying the *CtDGAT2b* gene and wild-type cells without any plasmid were grown in media devoid of any free fatty acid or containing oleic acid of different concentrations. In media lacking free fatty acids, both wild-type and QM cells exhibited normal growth, but the QM strain started showing cytotoxic effect with the addition of 0.025 mM oleic acid in the medium (Figure 5A). When the concentration of oleic acid in the medium increased to 0.5 mM, the growth of QM cells was arrested due to toxicity, but wild-type yeast cells continued to grow with little cytotoxic effect. However, upon overexpression of the CtDGAT2b enzyme, the growth of QM cells was rescued at the critical oleic acid concentration, which was found to be toxic to the QM cells with or without the non-recombinant plasmid (Figure 5A).

**Figure 5:** Enzymatic activity of CtDGAT2b in *S. cerevisiae* QM strain rescues the yeast cells from the cytotoxic effect due to free fatty acid in growth medium. (A) Growth rescue of transformed QM cells in oleic acid containing media. Yeast nitrogen base media was used for the growth of wild-type (WT) and non-transformed QM cells with dextrose and uracil, whereas raffinose and galactose with no uracil was used for the QM transformant (QM-pYES2 or QM-CtDGAT2b) to induce the expression of transgene. Two microliters of yeast cells (O.D. 1), after serial dilutions (10^−1^, 10^−2^, 10^−3^, 10^−4^ and 10^−5^) were spotted on solid media without or with 0.025 mM and 0.5 M oleic acid. (B) Growth phenotype of QM cells harboring non-recombinant plasmid pYES2 (QM-pYES2) and recombinant plasmid with the *CtDGAT2b* gene (QM-CtDGAT2b) on solid media supplemented with three different fatty acids- α-linoleic acid (C18:3), arachidonic acid (C20:4), erucic acid (C22:1) after 4 days at 30°C. (C) Fatty acid composition of TAGs isolated from the wild-type yeast (WT) and transformed QM cells (QM-CtDGAT2b) grown in liquid media (i) without any free fatty acid, and supplemented with (ii) α-linolenic acid (ALA), (iii) arachidonic acid (ARA) and (iv) erucic acid (EA).

It is known that lipid bodies are present in the wild-type *S. cerevisiae* cells, and completely absent in the QM strain. To assess whether the cells rescued from free fatty acid toxicity actually form lipid bodies, QM cells transformed with the non-recombinant plasmid or recombinant plasmid carrying the *CtDGAT2b* gene were visualized by confocal microscopy after Nile red staining. The analysis revealed cytoplasmic lipid droplet formation in QM cells transformed with the recombinant plasmid, but no such lipid bodies were found in cells transformed with the non-recombinant plasmid (data not shown). From these findings, it is evident that the CtDGAT2b isozyme is efficient in mobilizing the free fatty acid pool into storage lipids.

To find out whether other unsaturated fatty acids, besides oleic acid could be incorporated into TAG of QM yeast cells upon expression of the CtDGAT2b, we compared growth phenotype of QM cells transformed with the non-recombinant plasmid and those with the recombinant plasmid carrying the *CtDGAT2b* gene on solid media supplemented with different fatty acids, like α-linolenic acid (ALA), arachidonic acid (ARA) and erucic acid (EA). After 4 days of incubation at 30°C on solid media, it was revealed that QM cells transformed with the *CtDGAT2b* gene grew successfully on solid media supplemented with different fatty acids than QM cells without the gene of interest (Figure 5B).

To verify any preference for specific fatty acid to incorporate into TAG by acyltransferase activity of CtDGAT2b, the QM cells with the gene and the wild-type cells without the gene were grown in liquid media supplemented with or without the above mentioned three exogenous fatty acids i.e., ALA, ARA and EA as these are not naturally present in yeast cells. In the absence of supplementary fatty acid, the recombinant CtDGAT2b formed TAG by utilizing endogenous fatty acids, and showed a clear preference for saturated C16:0 and C18:0 fatty acids as compared to the endogenous ScDGAT of wild-type yeast, which was more selective towards monounsaturated C16:1 and C18:1 acyl species [Figure 5C (i)]. Thus, TAGs formed by the activity of CtDGAT2b are substantially more saturated than those formed by the wild-type ScDGAT. In three fatty acid supplementary experiments, the same trend of endogenous fatty acid utilization specificity was observed for TAG formation by both the recombinant CtDGAT2b and the wild-type ScDGAT. With respect to the exogenous fatty acid utilization, the wild-type ScDGAT showed more preference towards supplemented ALA during TAG formtaion compared to the recombinant CtDGAT2b yeast cell [Figure 5C (ii)], whereas the opposite selectivity was observed in case of ARA or EA supplementation [Figure 5C (iii, iv)].

Few reports documented on the substrate specificity of DGAT2 enzymes in the past [6]. The *V. fordii* DGAT2 showed preferential incorporation of α-eleostearic acid in TAGs of seed [17]. On the contrary, the DGAT2 enzyme of castor bean and *Vernonia galamensis* displayed higher selectivity for substrates containing ricinoleic and vernolic acid, respectively [18], [41]. Among the fungi, the *Mortierella ramanniana* DGAT2 showed enhanced activity towards medium-chain fatty acyl-CoAs, like myristoyl-CoA [42], whereas the DGAT2 of yeast *S. pombe* was found to prefer palmitic acid over oleic acid [43]. In our present study, we observed that the CtDGAT2b has substrate selectivity more towards saturated than unsaturated acyl species in heterologous yeast expression system. This has definite correlation to our earlier report and well justifies the fact that the oleaginous *C. tropicalis* natural isolate SY005 is capable of producing storage lipid enriched with saturated fatty acids, particularly stearic acid.

### Lipid productivity efficiency of CtDGAT2b in heterologous yeast system is affected by deletion, insertion or replacement of amino acids in five exclusive regions other than the highly conserved DGAT-specific motifs

Since two CtDGAT2 isoforms are unique with respect to the presence of five additional stretches of amino acids i.e., D1 to D5 compared to other reported DGAT2 proteins (Figure 1B), mutagenesis analyses were carried out within these domains to understand the detailed functions of these novel acyltransferases. Among the two functionally active isozymes, since the CtDGAT2b is capable of yielding more TAG compared to CtDGAT2a in heterologous expression system, the former was selected as candidate gene for in-depth analysis. For this investigation, initially 5 deletion genetic constructs were prepared in addition to the full length CtDGAT2b isoform. Subsequently one more deletion, one insertional and two replacement mutant gene constructs were prepared.

Firstly, to verify whether the 5 deleted gene constructs (Figure 6A, B) do indeed encode a protein with DGAT activity, transformed QM cells were grown as usual to check for cell morphology and induced by galactose to observe for the expression of recombinant protein. Analysis revealed that the 5 deleted gene constructs i.e., ΔD1, ΔD2, ΔD3, ΔD4 and ΔD5 along with the full length CtDGAT2b upon transformation into QM yeast cells showed no alteration in cell growth morphology (Figure 6C), and resulted in the expression of expected size recombinant protein, as depicted for few samples (Figure 7C). Subsequently, formation of lipid bodies in transformed QM cells was monitored through Nile red staining followed by confocal microscopy (Figure 7A). Among the five deleted constructs tested, trace amounts of TAGs were detected in the QM cells expressing the deleted genes ΔD1(1–21), ΔD4(341–384) and ΔD5(481–571); whereas those expressing ΔD2(170–187) and ΔD3(252–271) variants showed significant amount of TAGs inside the cells (Figure 7A).

**Figure 6:** Deletion mutagenesis of the *CtDGAT2b* gene followed by the expression of each mutated version in *S. cerevisiae* QM strain. (A) Schematic diagram of the five deletion mutants- ΔD1 to ΔD5 of the full length *CtDGAT2b* gene corresponding to the five unique stretches of amino acids represented as D1 to D5 in Figure 1B. (B) Ethidium bromide-stained 1.2% agarose gel showing restriction enzymes (*Bam*HI+*Eco*RI) digestion profile of the recombinant pYES2 plasmid carrying either the full length *CtDGAT2b* gene or each of the five deleted versions of *CtDGAT2b* gene. (C) Growth pattern of QM yeast cells transformed with the individual gene construct carrying either the full length *CtDGAT2b* or each of the five deletion mutants, after 4 days of plating of yeast cells (O.D. 1) in different dilutions (10^−2^ to 10^−5^).

**Figure 7:** Differential enzymatic activity of various mutated versions of the CtDGAT2b towards TAG formation in *S. cerevisiae* QM strain. (A) Nile red fluorescence confocal microscopy showing lipid body formation is restored in yeast QM cells albeit at different extent, upon expression of five deletion mutants of CtDGAT2b. (B) Differential complementation of the TAG-deficient phenotype of the yeast QM strain by enzymatic activities of five deleted constructs ΔD1(1–21), ΔD2(170–187), ΔD3(252–271), ΔD4(341–384) and ΔD5(481–571). Neutral lipid fractions were separated by TLC, and lipid spots were visualized as described in experimental methods. (C) Western blot showing the recombinant proteins of 60–63 kDa produced upon galactose induction of yeast QM cells transformed with the recombinant pYES2/CT plasmid carrying either the full length *CtDGAT2b* gene or the mutant ΔD4(341–384) or ΔD6(365–374) version. Immunodetection was carried out with mouse anti-His monoclonal antibody. (D) Schematic diagram showing the insertion and replacement of amino acids at a unique polyglutamic acid stretch of ten residues in the segment ΔD4(341–384) created mutants D7(364::365–376), D8(364::KKKKKKKKKK) and D9(364::AAAAAAAAAA). (E) Bar and line diagrams representing gravimetric measurement and Nile red fluorescence assay of lipid content in QM cells after expression of the full length CtDGAT2b and all the five deletion, one insertional and two replacement mutants; along with the WT and QM cells transformed with the non-recombinant plasmid as positive and negative controls, respectively. Fluorescence was measured at the stationary phase using 485nm (excitation) and 540 nm (emission) before and after the addition of Nile red dye, and expressed in arbitrary unit.

Further, to quantify the differential lipid accumulation, total lipid extracts from transformants were analyzed by thin layer chromatography (Figure 7B), and lipid contents were estimated by Nile red fluorescence spectrometry assay (Figure 7E). Analyses revealed that the deletion of D1 segment of amino acids (1–21) at the N-terminal region of the protein, resulted in an enzyme with less than 64% of activity compared to the full length CtDGAT2b as reflected by TAG content of transformed cells (Figure 7E). Among the other segments, D2(170–187) and D3(252–271), being located in the middle region displayed a little decrease of enzyme activity ∼34% and ∼23% respectively, in TAG accumulation compared to the CtDGAT2b. On the other hand, the deletions of the segment D4(341–384) located in the middle region and the segment D5(481–571) situated at the C terminal region of protein resulted very significant decreases in enzyme activity, as reflected by 76% and 88% decrease in TAG accumulation, respectively compared to the full length CtDGAT2b (Figure 7D). These findings indicate that the hydrophilic regions at the middle and C-terminal tail of CtDGAT2 are more sensitive to any alteration than N-terminus in terms of enzyme activity. Another interesting inference from these results is that the deleted segment D4(341–384), being located in the middle part of the CtDGAT2b with three predicted phosphorylation sites (Table S1) and carrying an unique glutamic acid stretch of 10 residues could play a critical role in enzyme activity. To further verify the importance of this repeat of glutamate, we created yet another deleted gene construct ΔD6(365–374) to exclude this repeat of gutamic acids (Figure 7D). Interestingly, the deletion mutant ΔD6(365–374) resulted a similar decrease of about ∼70% in enzyme activity (Figure 7E) compared to the full length CtDGAT2b, implying that the whole D4(341–384) segment is not accountable for the critical enzyme activity, rather a specific deca-glutamic acid stretch is more imperative, and this repeat sequence has positive effect on the enzyme activity. As mentioned earlier that the CtDGAT2b is capable of yielding 12.5% more TAG compared to the CtDGAT2a isozyme in QM yeast cells (Figure 4) and it naturally possesses a repeat of 10 glutamic acids compared to that of eight glutamic acids in CtDGAT2a exactly in the same position of the polypeptide (Figure 1B). In the context of these findings, we hypothesized that the insertion of extra glutamic acids in this region might have more positive effect on the enzyme activity. Thus, we incorporated additional two glutamic acids in CtDAT2b to make a stretch of twelve glutamic acids in this region from residue 365 to 376 at position 364, creating one insertional gene variant, D7(364::365–376) (Figure 7D). Surprisingly, this insertional mutant showed an increase of more than 40% in enzyme activity compared to the full length CtDGAT2b (Figure 7E), resulting in the creation of a hyperactive mutant version of CtDGAT2.

To examine further whether this enhanced acyltransferase activity of CtDGAT2b is specific to only negatively charged amino acid repeat in this position, we inserted a stretch of 10 lysine (K), a positively charged amino acid in place of negatively charged glutamic acid (E) at the same position to make the first replacement gene variant, D8(364::KKKKKKKKKK) (Figure 7D). In contrast to D7 variant, this mutant D8 resulted a decrease in enzyme activity of about ∼80% compared to the wild-type CtDGAT2b (Figure 7E), suggesting the augmentation effect on the enzymatic activity in D7 variant was sequence specific to glutamic amino acids. We had also replaced the naturally occurring 10 glutamic acids in CtDGAT2b by 10 residues of alanine (A), a nonpolar and nonreactive amino acid that doesn't generally play major role in protein function, at the same position (Figure 7D). In comparison to D7 and D8, this second replacement gene mutant D9(364::AAAAAAAAAA) caused ∼40% decrease in the activity of enzyme with respect to the full length CtDGAT2b (Figure 7E).

Previously, site-directed mutagenesis on the conserved motifs of *S. cerevisiae* DGAT2 revealed the functional role of this enzyme and topological orientation of the DGAT2-specific signature motifs [33]. Similar kind of studies carried out on the signature motifs of *S. cerevisiae* DGAT1 demonstrated that the mutagenesis of His-426 to alanine impaired the ability of DGAT1 to synthesize triacylglycerols [44]. Among the plant species, mutagenesis experiment was conducted on the signature regions putatively involved in enzyme function or regulation of DGAT1 of *Tropaeolum majus* [40].

The present mutagenesis study for the first time provides evidence that the additional non-conserved domains are very crucial in the regulation of DGAT2 enzyme, besides the highly conserved DGAT-specific motifs. Recognizing the essential role of highly conserved DGAT2-specific motifs, we have documented that the additional five domains (D1 to D5) of CtDGAT2 play vital function in influencing the acyltransferase activity in the *C. tropicalis* SY005 strain for neutral lipid production. More importantly, the unique stretch of 10 negatively charged glutamic acid residues naturally present in CtDGAT2b participates a central role in the increased enzymatic activity compared to the CtDGAT2a, leading to the enhanced TAG accumulation in this oleaginous yeast strain. Additionally, a hyperactive version of CtDGAT2 enzyme with 12 glutamic acid residues has been developed and tested during the course of this study, in contrast to the naturally existing CtDGAT2a and CtDGAT2b having eight and 10 glutamic acid residues, respectively.

## Conclusions

We have cloned and functionally characterized two novel homologues of *DGAT2* gene from the oleaginous yeast *C. tropicalis* SY005 strain, which is a natural producer of enhanced storage lipid enriched with saturated fatty acids, particularly stearate. The two isozymes- CtDGAT2a and CtDGAT2b open up the scope for further investigation on the novel structure-function relationship in the repertoire of DGAT enzymes. It is worthy to mention here that the *C. tropicalis* SY005, which we have studied, is a natural isolate from the rhizospheric soil; but the pathogenic yeast *C. albicans* is responsible for the fungal disease, known as candidiasis in animals including human. Therefore, we are tempting to speculate that similar kind of structurally novel DGAT2 enzyme(s) may be present in the pathogenic yeasts or fungi, and could be the target to design drug molecules to selectively inactivate the TAG production, leading to the blockage in the life cycle of this organism. Additionally, the newly cloned *CtDGAT2b* gene or its hyperactive mutant version will be useful for the enhanced production of lipid feedstock in other organisms through metabolic engineering.

## Supporting Information

Figure S1 **Identification of an uncharacterized DGAT-like gene in** ***Candida tropicalis*** **genome sequence.** (A) Result of BLAST analysis within *Candida* group, using amino acid sequence of the YALIOE32769g protein of *Y. lipolytica* as input (query) sequence. The identified putative DGAT2 protein of *C. tropicalis* showing maximum identity with the query is indicated by black arrow. (B) The hypothetical protein shows the presence of domains specific for DGAT, LPLAT and MGAT superfamily protein.
(TIF)

Figure S2 **PCR-mediated cloning of the putative** ***DGAT2*** **gene from the oleaginous yeast** ***C. tropicalsis*** **SY005 strain.** (A) Ethidium bromide-stained 1.2% agarose gel showing the PCR amplified DNA fragment of *CtDGAT2* gene. Lane 1: PCR product; Lane 2: pUC18 DNA digested with *Hin*f1 as molecular weight marker. (B) Ethidium bromide-stained 1.2% agarose gel showing characteristic restriction enzyme digestion of the pTZ57R/T/CtDGAT2 recombinant plasmid with *Bam*HI (lane 2), *Xba*I+*Bam*HI (lane3), *Eco*RI+*Bgl*II (lane 4), *Bgl*II+*Pst*I (lane 5), *Bgl*II (lane 6), *Eco*RI (lane 7) and *Bam*HI digested pTZ57R/T vector (Lane1). Lane M: pUC18 DNA digested with *Hin*f1 as molecular weight marker.
(TIF)

Figure S3 **Alignment of the amino acid sequences of CtDGAT2a and CtDGAT2b isoforms.** The amino acid sequences were derived from the corresponding two homologues of *CtDGAT2* gene cloned from the oleaginous yeast *C. tropicalis* SY005 strain. Differences of residues between CtDGAT2a and CtDGAT2b isoforms are indicated by black-and-white over a yellow-background.
(TIF)

Figure S4 **A phylogram showing relationship of two CtDGAT2 isoforms with diverse hypothetical and characterized DGAT-like proteins of representative organisms from fungi including yeasts, algae, higher plants and animals including human.** The alignment was generated using ClustalW and the phylogram was constructed by the neighbor joining method with Mega 5.2 software. Different DGAT1s and DGAT2s from various organisms with respective GenBank accession numbers are as follows: AtDGAT1, *A. thaliana AAF19262*; BnDGAT1 *Brassica napus AAD45536*; CeDGAT1 *Caenorhabditis elegans AAF82410*; HsDGAT1, *Homo sapiens AAC37532*; MmDGAT1, *Mus musculus AAC72917*; NtDGAT, *Nicotiana tabaccum AAF19345*; PfDGAT, *Perilla frustescens AAG23696*; RcDGAT1, *Ricinus communis AAR11479*; AcDGAT2, *Ajellomyces capsulatus XP_001540241*; AtDGAT2, *Arabidopsis thaliana* NP_566952; AcDGAT2, *Aspergillus clavatus XP_504700.1*; CrDGAT2a, *Chlamydomonas reinhardti XP001702848*; CrDGAT2b, *C. reinhardti* XP_001691447; CrDGAT2c, *C. reinhardti XP_001694904*; CrDGAT2d, *C. reinhardti XP_001693189*; CrDGAT2e; *C. reinhardti XP_001701667*, HsDGAT2, *Homo sapiens AAK84176*; MrDGAT2a, *Mortierella ramanniana AAK84179*; MrDGAT2b, *M. ramniana AAK84180*; MmDGAT2, *Mus mulus AAK84175*; OtDGAT2 *Ostreococcus taurii CAL58088*; RcDGAT2, *Ricinus communis XP_002528531*; ScDGAT2, *Saccharomyces cerevisiae NP_014888*; SpDGAT2, *Schizosaccharomyces pombe XP_001713160*; VfDGAT2, *Vernonia fordi ABC94474*; YlDGAT2, *Yarrowia lipolytica XP_504700.1*.
(TIF)

Figure S5 **TMHMM prediction for transmembrane domains of two CtDGAT2 isoforms.** Two CtDGAT2 isoforms have same internal structure. One potential transmembrane helix present at amino acid position 91–113. Blue circle indicates the higher probability for transmembrane regions in CtDGAT2b isoform between the residues 220–300 compared to CtDGAT2a.
(TIF)

Table S1 **Putative functional motifs of two CtDGAT2 isoforms predicted by PROSCAN.**
(DOC)

Table S2 **List of primers used in this study.**
(DOC)
